The article "A Survey Research on the Willingness of Gynecologists to Employ Mobile Health Applications" was retracted in 2023. Reasons: signs of a paper mill; suspected computer-generated content; unreliable results or conclusions; concerns about the data.

# A Survey Research on the Willingness of Gynecologists to Employ Mobile Health Applications

**DOI:** 10.1155/2021/1220374

**Published:** 2021-12-31

**Authors:** Malik Bader Alazzam, Ahmad Tawfig Al-Radaideh, Raed Ahmed Alhamarnah, Fawaz Alassery, Fahima Hajjej, Azmi Halasa

**Affiliations:** ^1^Faculty of Computer Science and Informatics, Amman Arab University, Amman, Jordan; ^2^Department of MIS, College of Business, Jadara University, Irbid, Jordan; ^3^Computer and Information System Department, University of Almaarefa, Riyadh, Saudi Arabia; ^4^Department of Computer Engineering, College of Computers and Information Technology, Taif University, P.O. Box 11099, Taif 21944, Saudi Arabia; ^5^Department of Information Systems, College of Computer and Information Sciences, Princess Nourah bint Abdulrahman University, P. O. Box 84428, Riyadh 11671, Saudi Arabia

## Abstract

In gynecological care, mHealth (mobile health) technology may play an important role. Medical professionals' willingness to use this technology is the key to its acceptance. Most doctors utilize mobile health technology; however, there is still room for improvement in the use of mHealth. Gynecologists were asked to participate in this research to see how open they were to use mobile health technologies. In this descriptive-analytical investigation, the researchers determined the average scores for each variable. The overall mean for preparedness to embrace mobile medical technology is 1.8 out of 2, as shown in Table 1. When it came to their desire to embrace mobile health technology, doctors' years of experience correlated negatively with their age. According to our findings, the amount of interest in mobile health technology is high. Patients' private information must be protected throughout the usage of this technology though. Mobile health technology may effectively reach patients in remote areas, but it is not a substitute for face-to-face encounters with medical professionals.

## 1. Introduction

There are around 59 million healthcare employees in the globe, and according to one forecast, the need for health workers would increase to 80 million workers by 2030 [1]. There is a paucity of hospitals and specialty workers, clinical access to healthcare, and weak interaction between doctors and patients, particularly in rural regions. To close this gap, healthcare staff must go down a long and time-consuming route, which is not without its challenges. It is described as the use of all telecom equipment, including handy smart devices, to satisfy the demands of patients providing information services related to the field of healthcare (mHealth) [1, 2]. World Health Organization (WHO) approved “mobile health” as a term for smartphone-assisted public health departments and medical, medical monitoring systems, personal digital assistants (PDA), and other electronic tools. In addition to monitoring healthcare progress, distributing educational materials, receiving tailored signals and support, and adopting self-management therapies, digital healthcare technology may be useful for a range of other applications. mHealth has the potential to play a key role in removing geographical barriers to the delivery of healthcare, as well as giving the possibility to provide health services to everyone, everywhere, or at any time in the world [1].

For healthcare practitioners to be able to offer high-quality treatment, they must have access to critical information about patients' historical and present medical problems. In order to transmit data and vital information, people are increasingly turning to mobile phones. As a result of the increased use of cell phone technologies, the exchange of information among both health providers and patients can be more efficient, it has the potential to be a successful technique for diseases' control and prevention. It can also be a promising strategy for improving the public welfare, particularly, for susceptible populaces by reducing inequalities in healthcare and improving public welfare [1, 3].

Furthermore, doctors and other professionals in healthcare have a positive outlook on health and digital healthcare technologies, according to prior polls. Many of these experts are eager to embrace this technology. Women with gynecological problems and illnesses may benefit from mobile health, according to a number of studies. However, there are several roadblocks in the way of putting such technology into practice. These impediments are either organizational in nature or are connected to stakeholders. Healthcare practitioners' reluctance to new technologies and methods is one of these hurdles to the use of this technology. The use of health information technology by healthcare professionals is critical to the field's long-term success. The desire of patients and healthcare practitioners to employ this technology determines the degree of acceptability of this technology. To prevent the loss of mHealth digital innovations, it is essential to study the degree of acceptability and desire to use these health apps from the beginning of their creation. Because of this, this study was conducted to evaluate how eager gynecologists are to use mHealth technology [4].

## 2. Areas of mHealth Applications

When considering health apps, it is important to examine the user's perspective as well as the features provided, medical specializations, and public health sectors in which they are employed [3, 5].

Universal healthcare and public health, according to this paper's authors, are best served by the use of mobile technology in several areas:

- Environmental factors
- Epidemiological phenomena
- Illness progression
- Therapeutic support

With this paper's authors, the most important mobile health and public health activities are as follows.

In order to demonstrate the potential of the mHealth field and to systematize existing knowledge, Sloninsky et al. (2017) conducted a study of previously referred material. mHealth applications are being developed in areas. Many of these include assistance for clinical decisions in the care setting, detection systems and clinical services, and support for health, including health promotion and community mobilization monitoring and reporting, [4].

Other mobile technologies that may be used for mHealth include smartphones, communication devices and cellphones, equipment for monitoring patient conditions, mobile healthcare equipment that provides remote treatment, and smartphones that can be used on the go [6]. This paper, published in 2011, provided the findings of a globe survey on eHealth, highlighting six activities carried out with the use of mHealth systems. These activities include communications with healthcare facilities (such as call centers and helplines), Health care institution-to-patient communication (such as adherence to medication recommendations, mementos of consultations, community mobilization, and raising health-related awareness), healthcare professional-to-healthcare professional communication, and intersectoral communication between healthcare professionals, for example, e-mail and instant messaging.

## 3. Empirical Evidences

Thus, the health and well-being of family caregivers have attracted widespread attention. Mobile health technology has been shown to deliver flexible and time- and cost-sparing interventions to support family caregivers across the care trajectory. Mobile health technology (mHealth) is “medical and public health practices supported by mobile devices, such as mobile phones, patient monitoring devices, personal digital assistants, and other wireless devices.”

Among the wireless technology used for mHealth interventions, short message service (SMS) and mobile health apps are deployed most frequently. Mobile health apps can promote self-care management. When conducting a comprehensive study to determine the efficacy and efficiency of mobile health technology in improving care and well-being services, we advocate categorizing mobile treatments into those that target certain populations, according to Free and colleagues. Mobile apps that gather information would be of particular interest to researchers in the field of healthcare, per the division. In addition to these apps, healthcare practitioners may make use of solutions that facilitate education and provide access to medical records, among other features. These include apps that allow for the transmission of diagnostic test results, monitoring illness progression, and decision-supporting tools. Both medical professionals and patients may benefit from such applications [4].

Patient-focused applications include those that allow appointment reminders to be sent, those that help establish a treatment plan, those that assist in the management of chronic illnesses, and those that encourage patients to comply with drug regimens. In order to assist behavior adjustment, patients and members of a particular group may make use of apps that help them cope with unexpected health situations, such as those needing first aid or presenting a health hazard [7]. Mobile apps make it feasible to target campaigns with health promotion aims to the whole population via the use of smartphones and other handheld devices.

Based on a study of publications that describe the findings of research on the influence of mobile phone apps on health outcomes, Fiordelli et al. (2014) conducted a systematic evaluation of the development of new applications for mobile phones. The authors focused on publications published between 2002 and 2011 that reported on the outcomes of testing mobile apps. A number of publications passing review requirements climbed from one to thirty, with the most popular, 63.2 percent, being mobile apps intended and the need for care in the event of chronic conditions, according to the results; 18.8 percent of apps supported preventative activities and the well-being of users, while 17.9 percent of reports were appropriate in emergency circumstances [8–11].

There were 20.5 percent of papers covered by this review that contained results from testing applications for diabetic patients, 13.7 percent that contained results from testing applications for the management of obesity and overweight, 12.8 percent that contained results from testing applications for mental health, and 8.5 percent that contained results from testing applications for helping people quit smoking. An overview of mobile features was also included in the evaluation. According to the researchers, among the apps, text messages were utilized in 49 percent, while custom functionalities for particular illnesses and health concerns were used in 32 percent. Using devices that work in conjunction with mobile phones (referred to as “add-ons”), for example, checking blood glucose levels or tracking physical activity, 12 percent of the applications were completed. Only 10 percent of respondents utilized voice calls, while 6 percent used video transmission and 3 percent used multimedia messaging. They also identified seven major areas of influence of the evaluated mobile applications, which were further subdivided. When it comes to illness management, the vast majority of applications (38 percent) were geared at achieving the advantages of health promotion and independence (33 percent). Applications were utilized less often for communication enhancement (22%), monitoring systems (21%), and data collection (21%) than for enhanced collaboration (20%), training and education (20%), and other purposes (13 percent) [12, 13].

Mobile phones and tablets are being increasingly integrated into the daily lives of many people worldwide. Mobile health (mHealth) apps have promising possibilities for optimizing health systems, improving care and health, and reducing health disparities. However, healthcare apps often seem to be underused after being downloaded. In a similar vein, Ali et al. (2020) reported three years later and undertook a review to assess the progress and current state of mHealth research, but less strict criteria were used. The examination covered further works released during the months of January and December of 2015. Up to 515 papers were included in the analysis as a consequence of this process. Three stages have been identified by researchers in the area of mHealth applications. The first, which lasted from 2006 to 2006, was dominated by PDA devices; furthermore, it also lasted from 2007 to 2012 and had also been controlled by basic mobile telephone functions; the third, which also would last from 2012 to the current time, was dominated by smart devices. Health promotion, illness prevention, diagnosis, treatment, monitoring, and assistance of health services were highlighted as the six primary aims of mobile interventions. For example, 51.5 percent of mHealth apps were developed to assist healthcare services, while 33.3 percent were developed to monitor healthcare services [14–16].

During this time span, none of the applications that were created had anything to do with health promotion or illness prevention. The majority of applications (30.1 percent) and health care assistance were for monitoring during the second period (25.9 percent). Preventive medicine accounted for just 10.9 percent of the applications, compared to 17.1 percent for diagnostic tests, 16.1 percent for medication, and 17.1 percent of applications for preventative medicine. Goal-oriented applications provide health services and those that monitor health continue to dominate the ultimate developmental stage of mHealth apps. National prevention applications, on the contrary, have climbed to 14.2 percent of all applications in the last year. Fifty seven percent of mobile applications pertinent to disease nations or health situations were developed after 2012, during the most recent period of mHealth development, with only 11.1 percent of applications related to infectious diseases and 14.5 percent of applications that were not targeted to a particular type of disease. When it comes to the technologies that were employed in this last stage of mHealth development, 48.4% of apps were loaded on a mobile device, 19.7% on an SMS device, 6.2 percent on automatic sensors, and 4.5 percent on different kinds of telephone communication and video conferencing. Using a mobile device to capture, show, analyze, and/or transmit medical photos and video content was found to be effective in 9.7 percent of solutions tested [14].

Wearable gadgets are among the most promising of today's technology [17]. Apart from its usage for communication, entertainment, and commercial operations, preventive care and public health are the primary areas of use for these technologies. According to how they are worn, wearable gadgets may be categorized into two categories. In terms of head-mounted wearables, we can think of things like head phones, sport activities or production helmets with headsets that include microphones, GPS locations, and displays, contact lenses with blood glucose sensors, glasses that display hardware and software interfaces installed in smartphones, and even transplanted microphones known as “throat tattoos” that offer voice commands. One of the most popular places to wear electronic devices is on the wrist or forearm. You can wear voice-activated computers on your wrist, check your physical activity with apps like running trackers, and track your GPS location using wearable electronics such as watches. Among the other options, there are implanted subcutaneous RFID sensors, which may be used for a variety of tasks such as unlocking doors, purchasing, and accessing computers. It is now possible to adapt wearable technological devices for specialized uses to each portion of the human body, which is a significant advancement in terms of practicality. Ingesting devices, which have been in use for many years in the field of gastroenterology diagnostics, might potentially be considered as wearable objects [18, 19].

## 4. Materials and Methods

The current analytical study was carried out in the year 2019. Gynecologists from Jordan were included in the study as participants. Using the Cochran formula, a sample size of 95 individuals was calculated, which after accounting for a 20% dropout rate, resulted in a final sample size of 100 participants. The simple random method was used to select participants from among the gynecologists at two different hospitals. All professionals had been using at least related applications, including health applications, and so as a result, they had a sufficient amount of knowledge about mobile health applications to share with their colleagues.

To gather data, the researchers devised a questionnaire based on findings from previous studies. This survey was divided into two parts [20]. The survey was divided into two sections; the first asked general demographic questions and the second asked about group members' readiness to use cellphone medical advances (or not). A three-point Likert scale was used in the development of the survey items (disagree, neutral, and agree). Five experts were surveyed to test the survey's validity, and the results of their responses were used to make revisions to the questionnaire. Cronbach's alpha was used to determine the reliability of the questionnaire [21].

The questionnaires were given out to the gynecologists who had given their verbal consent to participate in the research. In the presence of the researcher, they completed the survey questionnaire. If the physicians felt that they needed more time, the questionnaire forms would be collected at a later date. Out of the 116 questionnaires sent, 92 were returned. Results were analyzed using the following scoring system: 0, 1, and 2 were used to indicate agreement or disagreement. IBM SPSS for Windows, version 26.0, was used to evaluate the data, which included summary analysis (frequency and mean scores) and inferential statistics (statistical significance). Percentage scales were used to assess people's desire to utilize mobile health: 0–20 percent indicated low, 21–40 percent indicated low, 41–60 percent indicated medium, 61–80 percent indicated good, and more than 80 percent rated outstanding.

## 5. Results

Table 1 and Figure 1 display the profile of the sample in terms of frequency distribution, with 88 gynecologists included. Ninety two percent of the physicians who took part in the study were female, and almost all of them had a cellphone (100 percent).

According to the findings, the average age of the doctors who took part in this research was 45.05 6.58 years old, with the lowest and highest ages being 32 & 55 years old, correspondingly. Aside from that, doctors had an average of 12.45 years of experience, which was 5.77 years less than the national average.

Table 2 depicts the willingness of gynecologists to employ mobile health technology in their practices. For mobile medical technology adoption, the total mean is 1.8 out of 2 in this table (79.12 percent of the total potential score). A mean of 1.79 out of 2 (89.5%) was rated a good score for this group's desire to employ mobile health technology, based on their own self-reports.

There was a statistically significant negative link seen between the average age and willingness of participating doctors to adopt digital health technologies (*P*=0.001 and *R* = 0.543) in the study. Younger physicians were more inclined to use digital healthcare technology in their offices than their older counterparts. There was also a correlation (*P*=0.001 and *r* = 0.498) between the number of years of professional experience that the physicians had and their intention to use mHealth technologies.

Gender did not have an effect on overall desire to use mHealth technologies (*P*=0.754), according to the independent *t*-test results (*P*=0.848).

## 6. Discussion

Gynecologists are eager when using digital healthcare technology, and the great majority of them assume that it can help them provide better care to their patients. However, the current study found that there are already concerns about how secure mobile phone apps are when it comes to patients' personal information [22].

### 6.1. Possibility of Using mHealth

Over two-thirds of the respondents to this poll said they were interested in using mobile health technologies to improve patient care. Our previous research has shown that using mHealth applications and mobile phones was both acceptable and comforting for patients as well as caregivers. Moreover, the results of a recent research revealed that the majority of patients are using cellphones, which is consistent with current findings. There are several necessary platforms to install and utilize mobile health technologies for both doctors and patients, and it seems that these platforms are widely available [23]. As seen in the graph, participants' desire to utilize this technology decreased significantly with increasing age. A number of similar studies have shown that age plays a significant role in the adoption of mHealth technologies and that, as one's age grows, the degree of acceptance of this technology diminishes. The findings of research by Guo et al. (2018) show that apparent personalization among teen users may enhance the adoption of apps. The acknowledgment of mobile health technology was found to be significantly influenced by factors including effort expectation, behavioral control, social influence, and favorable settings which were shown to be relevant in the research by Hoque and Sorwar (2018).

There will be a rise in the use of phone apps among older people whether they are created in such a way that their use has a positive influence on the job or that they are simple to use, and there is a positive public mood in favor of the new technology and infrastructure. Older people's fear of technology and reluctance to change seems to be the most significant factor affecting older people's adoption of digital health technology [24]. This can be complicated by the fact that retired generations are less talented and self-efficient with using emerging technologies compared to younger people [25]. First, it is advised that mobile medical technology apps be built as designs and offered as trial runs so that users may review the usability of the programmed and submit concerns to the designers. This will help promote acceptance of mobile medical technology among older people. Additional training hours for older persons are needed to alleviate their technical anxiety and apprehension about implementing new technology and ongoing help after the modern technology is in place.

## 7. Conclusions

It was found that 89.5 percent of respondents said they were excited about adopting mobile health technology in their practices. They considered it a beneficial tool for improving the health of their patients and boosting the efficacy of their own practices. However, several patients expressed concerns regarding the security of their personal information when using mHealth technology. These gynecologists also believe that while office visits cannot yet be replaced by mobile health technology, it is an excellent choice for providing treatments to those who live in remote places in which affordable healthcare is challenging, and it may help to establish unity in the healthcare system [25]. MHealth development environment should take place on a secure and safe infrastructure that adheres to the security procedures in a virtual network, according the authors of this paper. In addition, doctors may find it comforting to realize that the accessibility of this technology benefits them rather than causes them problems. As a result of this, the development team must begin by including the opinions of doctors into the software development process. We propose looking at the willingness of other healthcare professionals to use this software and any extra infrastructure needed to encourage the use of advanced technologies by healthcare providers [4].

## Figures and Tables

**Figure 1:** Demographics of the study.

**Table 1:** Demographics of the study.

Variables	Groups		
Gender	Female	88	92.63157895
	Male	7	7.3684

Owning a cell phone	Yes (regular cell phone)	0	0
	Yes (smartphone)	95	100
	No	—	

Heard about “mobile health”	Yes	86	90.52631579
	No	9	9.473684211

**Table 2:** Mean and frequency of mobile health technology willingness.

	Agree	Neutral	Disagree	Mean score out of 2
A mobile phone is simple to use	95	0	0	2
	(100)	0	0	

Patients will benefit from having access to health services and consultations through their mobile phones	62	6	27	1.7
	(65.26)	(6.31)	(28.42)	

I would be interested in utilising it if it allowed me to answer patients' inquiries through mobile phone apps	68	3	24	1.7
	(71.57)	(3.15)	(25.26)	

I would be willing to substitute a phone call for a face-to-face visit if it meant I could better react to patients' inquiries	74	3	18	1.8
	(77.89)	(3.15)	(18.94)	

Patients' face-to-face appointments may be replaced by using mobile health technology, which has the potential to be just as beneficial	78	5	12	1.76
	(82.10)	(5.26)	(12.63)	

I am comfortable using a mobile phone to track the health of my patients	71	7	17	1.69
	(74.73)	(7.36)	(17.89)	

It is possible to remind patients of their medical instructions using mobile health technology	77	5	13	1.75
	(81.05)	(5.26)	(13.68)	

Mobile health technology allows me to make fast medication modifications for my patients when I need to	80	1	14	1.86
	(84.21)	(1.05)	(14.73)	

The usage of smartphones is essential in order to adhere to medical instructions	77	2	16	1.72
	(81.05)	(2.10)	(16.84)	

The use of mobile health technologies may help me build a strong connection with my patients so that I can better monitor their health	76	3	16	1.69
	(80)	(3.15)	(16.84)	

By using this technology, I will be able to work more effectively and efficiently	70	2	23	1.7
	(73.68)	(2.10)	(24.21)	

Patients' treatment procedures will be improved as a result of the use of this technology	69	5	21	1.6
	(72.63)	(5.26)	(22.10)	

Healthcare in distant and rural locations will be improved through the use of mobile health technologies	75	3	17	1.78
	(78.94)	(3.15)	(17.89)	

Health equality may be achieved by using this technology	72	4	19	1.77
	(75.78)	(4.21)	20	

Accountability of health information is protected when using mobile devices	70	7	18	1.69
	(73.68)	(7.36)	(18.94)	

Patients' treatment expenditures may be reduced by using mobile health	79	4	12	1.82
	(83.15)	(4.21)	(12.63)	

It is my belief that most patients will make use of this technology if it is made available to them	81	6	8	1.92
	(85.26)	(6.31)	(8.42)	

I intend to utilize this technology in the future	79	5	11	1.86
	(83.15)	(5.26)	(11.57)	

TOTAL	1353			1.81

## Data Availability

The data used to support the findings of this study are included within the article.
